The article "Knowledge, Attitude, and Practice regarding Narrative Medicine among Chinese Medical Personnel: An Online Cross-Sectional Survey" was retracted in 2023. Reasons: signs of a paper mill; compromised peer review; unreliable results or conclusions.

# Knowledge, Attitude, and Practice regarding Narrative Medicine among Chinese Medical Personnel: An Online Cross-Sectional Survey

**DOI:** 10.1155/2022/3329360

**Published:** 2022-10-12

**Authors:** Tong Guo, Yongli Sun, Guo Li

**Affiliations:** ^1^Beijing Tiantan Hospital, Capital Medical University, Beijing 100070, China; ^2^School of Medical Humanities, Capital Medical University, Beijing 100069, China; ^3^Beijing Fengtai Hospital of Integrated Traditional Chinese and Western Medicine, Beijing 100072, China

## Abstract

**Background:**

Narrative medicine has been applied as a model for humane medical practice in many countries. However, it was not introduced in China until 2011 and there has been no standardized assessment of Chinese medical personnel regarding their perception and application of narrative medicine-related theories. This study is aimed at investigating Chinese medical personnel's knowledge, attitude, and practice regarding narrative medicine and the factors that influence it.

**Methods:**

An online questionnaire based on the knowledge, attitude, and practice model was distributed among Chinese medical personnel from December 2021 to March 2022. All in-service medical personnel across China who had access to the Internet were eligible. Two independent samples *t*-tests, one-way analysis of variance, Pearson's correlation analysis, and multivariate linear regression were conducted for data analyses.

**Results:**

The participants' scoring rates for knowledge, attitude, and practice were 49.62%, 47.18%, and 41.43%, respectively. Significant influencing factors for knowledge were education level, religious belief, professional role, title, working years, and institution categories; those for attitude were education level, religious belief, professional role, and working years; and those for practice were professional title, religious belief, working years, and institution categories.

**Conclusions:**

Chinese medical personnel have generally good knowledge of, attitudes towards, and practice of narrative medicine; however, there remain deficiencies in their understanding of certain important concepts, their attitude towards narrative medicine, and the application of narrative skills in their daily work. Thus, to improve narrative medicine practice in China, the application of strategies based on theoretical, educational, and institutional aspects is warranted.

## 1. Introduction

Narrative medicine (NM), which is defined as the incorporation of narrative competence into the practice of medicine, was first proposed by Rita Charon in 2001, originated in the United States, and gained its popularity especially through the Medical Narrative Master's Degree Program of Columbia University. NM has since been applied in many countries as a model for medical humanism and effective medical practice [1, 2]. In China, however, NM was not introduced until relatively late, in 2011 [3]. Further, current doctor–patient relationships in China seem to be exceptionally strained, mainly as a result of shortages of medical resources and a growing demand for more personalized medical services [4]. This indicates the applicability of NM to the Chinese situation, as it has been found that NM can narrow the personal distance between doctors and patients, assist the effective treatment of patients and their families [1, 5, 6], and facilitate the provision of respectful, empathetic, and nurturing medical care [7–10]. Additionally, application of NM may mitigate the risk of burnout among medical professionals [11, 12]. However, despite NM's significance and possible advantages for relieving doctor–patient tension, literature on the recognition and application of NM in China remains limited, and there have been no similar standardized assessments of Chinese medical personnel regarding their perception and application of NM-related theories, which poses difficulty for the next-step policies on NM in China. In the present study, we conducted, using an online questionnaire, a cross-sectional survey of Chinese medical personnel in terms of their knowledge regrading, attitude towards, and practice of NM and also sought to determine the factors that influence such knowledge, attitude, and practice. In recent years, narrative educators have been advocating interdisciplinary cooperation in the field of narrative education, which involves students, educators, and facilitators with different professional background and encourages interdisciplinary communication from various angles [13, 14]. Therefore, we included not only doctors and nurses but also other members of Chinese medical system, including medical technicians, pharmacists, and hospital managers to explore from a multidisciplinary perspective beyond merely focusing on physicians, surgeons, and nurses. Our survey was based on the knowledge, attitude, and practice (KAP) model, which is an effective public-health tool that constitutes an easily applicable approach to determining individuals' knowledge and actions regarding a focus topic [15].

The article "Knowledge, Attitude, and Practice regarding Narrative Medicine among Chinese Medical Personnel: An Online Cross-Sectional Survey" was retracted in 2023. Reasons: signs of a paper mill; compromised peer review; unreliable results or conclusions.

## 2. Methods

### 2.1. Participants

All in-service medical personnel across China who had access to the Internet were eligible to participate in this online cross-sectional survey. The survey was conducted from December 2021 to March 2022. As a result of the Coronavirus Disease 2019 Pandemic, data were collected using the online questionnaire system Wenjuanxing (https://www.wjx.cn), which is widely used academically in China. The link for the questionnaire generated by Wenjuanxing was shared with eligible medical personnel via social-media platforms (e.g., WeChat). To reduce the risk of repeat submissions, IP-address-restriction technology was used. Prior to their commencement of the survey, all participants were informed of the study purpose and provided informed consent (through an online form). This study conformed to the guidelines of the Declaration of Helsinki and was approved by the Ethics Committee of Capital Medical University. All participants were assured of the anonymity and confidentiality of their responses and data, as well as their right to withdraw from the study at any time. Finally, a total of 2,145 participants completed the online questionnaire.

### 2.2. Questionnaire

Our questionnaire, which was entitled *Chinese Medical Personnel's Knowledge, Attitude, and Practices regarding Narrative Medicine*, was based on the KAP model [16] and Rita Charon's narrative theories [1, 2] and was developed and validated through expert review.

The questionnaire comprised the following four parts:

(1) Informed consent: this section included an introduction to the study, detailed the voluntary, anonymous, and confidential nature of participation, provided a guide for completing the questionnaire, and included an invitation to participate and an option to provide informed consent. Only participants who selected the “agree to participate” option could proceed to the next part of the questionnaire
(2) Participants' basic information: this section collected data regarding eight demographic variables, including gender, age, education level, marital status, and occupation-related information
(3) General cognition of NM: this section included four items, which measured participants' basic knowledge of NM, basic knowledge of parallel medical records, general comprehension of NM, and their usage of narrative methods in their daily work, respectively
(4) Knowledge, attitude, and practice regarding NM:
  - Knowledge of NM: this section comprised a nonscale part and a scale part, yielding a total of 15 items. The nonscale part (six items) focused on participants' knowledge of the difference between “disease” and “sickness” and on their knowledge of narrative relationships, narrative types, and parallel medical records. Participants could select one or multiple responses to these items. Meanwhile, the scale part (nine items) focused on participants' understanding of specific details regarding NM (e.g., effective tools for and purposes of NM). Each item in the scale was scored using a five-point Likert scale, with total scores ranging from 9 to 45. A lower total score or scoring rate (explained below) indicated better mastery of NM-related knowledge
  - Attitude towards NM: this section focused on participants' subjective feelings regarding NM (e.g., their attitude towards applying certain narrative behaviors) and featured a total of 11 items. Each item was rated using a five-point Likert scale, and total scores ranged from 11 to 55. A lower total score or scoring rate indicated a more positive attitude towards NM
  - Practice of NM: this section concerned the respondents' practical experience of NM, as well as their performance when practicing NM (e.g., their relationship with patients in their daily work); it featured a total of 12 items. Each item was rated using a five-point Likert scale, and total scores ranged from 12 to 60. A lower total score or scoring rate indicated better practice of NM

The article "Knowledge, Attitude, and Practice regarding Narrative Medicine among Chinese Medical Personnel: An Online Cross-Sectional Survey" was retracted in 2023. Reasons: signs of a paper mill; compromised peer review; unreliable results or conclusions.

### 2.3. Statistical Analysis

Data were analyzed using IBM SPSS Statistics for Windows, version 26.0 (IBM Corp., Armonk, N.Y., USA). Continuous variables were expressed as means ± standard deviations (*M* ± SD), while categorical variables were expressed using frequencies and percentages. The scoring rates for each option and item and the total scores for each KAP element were calculated by dividing the actual scores for the option, item, or total items by the total possible score for the option, item, or total items, respectively, and then multiplying this by 100%. For univariate analysis, two independent samples *t*-tests and a one-way analysis of variance (ANOVA) were conducted to compare participants with different demographic characteristics. Pearson's correlation analysis was used to explore correlations among the participants' KAP levels. For multivariate analysis, statistically significant variables were considered independent variables and then incorporated into the multivariate linear regression equation. Identical analyses based on 836 doctors' scores were also conducted since certain questions (such as those regarding writing medical records) may be more suitable for physicians and surgeons. *p* < 0.05 was considered to indicate statistical significance (two-tailed).

### 2.4. Validity and Reliability

The designed questionnaire was reviewed by several experts. Before the application of the formal survey, a pilot study was conducted to examine its reliability. The Cronbach's alpha coefficients for the KAP scales were 0.548, 0.743, and 0.883, respectively, all of which were acceptable.

### 2.5. Patient and Public Involvement

As a result of the nature of this study, which solely focused on medical professionals' knowledge, attitudes, and practices regarding NM, no patients or members of the general public were involved in the design, data submission, or data collection.

The article "Knowledge, Attitude, and Practice regarding Narrative Medicine among Chinese Medical Personnel: An Online Cross-Sectional Survey" was retracted in 2023. Reasons: signs of a paper mill; compromised peer review; unreliable results or conclusions.

## 3. Results

### 3.1. Participants' Demographic Characteristics

All completed questionnaires (*n* = 2,145) were advanced to the subsequent data analysis. The sample included respondents from various medical institutions across China (mainly from Beijing, Jiangsu, and Guangdong provinces). Most participants were female (1,214 [56.07%]), aged 30–50 years (1,305 [60.84%]), had a bachelor's degree or above (1,517 [70.72%]), were married (1,522 [70.96%]), were working as doctors or nurses (1,290 [60.14%]), had a primary title (e.g., resident physician) (821 [38.28%]), had been working for less than 20 years (1,619 [75.47%]), and were working in public medical institutions (2,114 [98.55%]; Table 1). Demographic characteristics of 836 physicians and surgeons are presented in Supplementary Table 1.

### 3.2. Participants' General Cognition and Basic Knowledge of Narrative Medicine

The results presented in Table 2 show that most participants had heard of the concept of NM (1,722 [80.28%]) and that their main sources of information were the Internet, lectures, conferences, etc. Nevertheless, relatively few participants were familiar with parallel medical records (1,633 [76.13%]), and only slightly over half of the participants were using narrative methods in their daily work (1,167 [54.41%]). Results of 836 doctors are presented in Supplementary Table 2.

With regard to basic knowledge of NM, most respondents were able to differentiate “disease” and “sickness” (1,631 [76.04%]); regarded the relationships between doctors and patients, as well as those among fellow medical professionals, as narrative relationships (1,497 [69.79%] and 1,530 [71.33%], respectively); and considered stories of doctor–patient contact and patients' as narrative types (1,661 [77.44%] and 1,477 [68.86%], respectively). However, only slightly more than one-third of the participants (783 [36.50%]) realized that parallel medical records are stories that describe doctor–patient contact. These results are also presented in Table 2, and those of 836 doctors are shown in Supplementary Table 2.

### 3.3. Scores for Knowledge, Attitude, and Practice regarding Narrative Medicine

The mean score for knowledge was 22.33 ± 4.87, with a total scoring rate of 49.62%. The highest and lowest mean item scores were 3.62 (“Shared decision-making among doctors and patients is not a practical way of implementing NM”) and 2.06 (“NM embodies the concept of patient-centered medicine”), respectively. The mean score for attitude was 23.42 ± 8.28, with a total scoring rate of 42.58%. The highest and lowest mean item scores were 3.66 (“I do not think practicing NM will have any effect on my medical practice”) and 2.03 (“I am willing to study NM-related courses”), respectively. The mean score for practice was 24.84 ± 8.98, with a total scoring rate of 41.40%. The highest and lowest mean item scores were 2.40 (“I try to write “medical confession stories” to alleviate my guilt regarding medical errors”) and 1.92 (“I am able to maintain good relationships with the patients I meet in my daily work”), respectively. These results are presented in Tables 3–5, respectively. Results of 836 doctors were similar to those of all the participants, which is shown in Supplementary Tables 3–5, respectively.

The article "Knowledge, Attitude, and Practice regarding Narrative Medicine among Chinese Medical Personnel: An Online Cross-Sectional Survey" was retracted in 2023. Reasons: signs of a paper mill; compromised peer review; unreliable results or conclusions.

### 3.4. Univariate and Multivariate Analyses of Factors Related to Knowledge, Attitude, and Practice Scores

Based on the results of two independent samples *t*-tests and a one-way ANOVA, statistically significant differences with regard to knowledge were observed between medical personnel with different ages, education levels, marital status, professional roles, titles, working years, and institution categories, respectively. Regarding attitude, significant differences were identified between medical personnel of different ages, education levels, professional roles, titles, and working years, respectively. Finally, for practice, significant differences were observed between medical personnel of different ages, education levels, professional roles, titles, working years, and institution categories, respectively. This meant that the same pattern of significant differences was observed for attitude and practice. These results are depicted in Table 1. Based on the results of Pearson's correlation analyses, the three elements of KAP were determined to be positively correlated with each other, with the strongest correlation being between attitude and practice (*r* = 0.805).

Multivariate linear regression analysis showed that significant influencing factors for knowledge were education level, professional role, title, working years, and institution categories. Regarding attitude, education level, professional role, and working years were significant factors. Finally, regarding practice, title, working years, and institution categories were identified as significant factors.

Longer working years predicted greater knowledge, a more positive attitude, and better practice. Medical personnel with higher education levels scored significantly better knowledge and attitude than those with lower education levels, and doctors had better knowledge and a more positive attitude than pharmacists, nurses, technicians, and managers. Finally, professional title was a positive predictor of knowledge and practice, and medical personnel in private medical institutions tended to have better performance in knowledge and practice. These results are also shown in Table 1.

The article "Knowledge, Attitude, and Practice regarding Narrative Medicine among Chinese Medical Personnel: An Online Cross-Sectional Survey" was retracted in 2023. Reasons: signs of a paper mill; compromised peer review; unreliable results or conclusions.

Results of univariate and multivariate analyses of factors related to the knowledge, attitude, and practice scores of 836 doctors exclusively are presented in Supplementary Table 1.

## 4. Discussion

As doctor–patient relationships in China are relatively strained, the dissemination and application of NM theories in Chinese clinical practice seem to be becoming increasingly necessary. Thus, in the present study we designed an online questionnaire based on the KAP model to comprehensively investigate Chinese medical personnel's knowledge, attitude, and practice regarding NM and to explore the factors that potentially influence their KAP in this regard. Notably, in contrast to the few previous assessments of Chinese medical personnel's engagement in NM [17, 18], the items in our KAP questionnaire were developed in a relatively standardized format, and there has been no similar KAP study regarding NM.

Overall, our online cross-sectional survey examined 2,145 medical personnel (including 836 doctors) across China and found that their KAP regarding NM is generally positive. To our knowledge, this is the first study to investigate the KAP of Chinese medical personnel regarding NM with no similar studies conducted before, and our findings have the potential to support the creation of strategies for developing NM in China.

### 4.1. Scores for the Knowledge, Attitude, and Practices regarding Narrative Medicine Questionnaire

The total scoring rate for knowledge was 49.62%, which is close to the “relatively agree” level. Item analysis showed that the mean scores for “NM embodies the concept of patient-centered medicine” (2.06) and “NM involves applying literary theories to medical practice” (2.12) were comparatively low, while the mean score for “Close reading and reflective writing are two NM tools” (2.24) was relatively high; this suggests that most participants had basic knowledge of the NM framework, but not of the specific methods or contents of NM. These findings indicate that future training programs should emphasize specific narrative skills and provide medical personnel with more opportunities to practice NM approaches they have learned.

The total scoring rate for attitude was 42.58%, which is also close to the “relatively agree” level. Item analysis revealed that the mean scores for “I am willing to study NM-related courses” (2.03), “I think cultivating narrative ability can improve my attention to and understanding of patients and also enhance my application of humanistic care” (2.06), and “I think an NM approach can provide patients with more personalized, humanized, and effective treatment” (2.06) were relatively low. The above data indicate that most Chinese medical personnel have a positive attitude towards NM; this has positive implications for the further promotion of NM in China.

The article "Knowledge, Attitude, and Practice regarding Narrative Medicine among Chinese Medical Personnel: An Online Cross-Sectional Survey" was retracted in 2023. Reasons: signs of a paper mill; compromised peer review; unreliable results or conclusions.

The total scoring rate for practice was 41.40%. Based on item analysis, the mean scores for “I am able to maintain good relationships with the patients I meet in my daily work” (1.92) and “I have sincere discussions with patients on a daily basis” (1.95) were comparatively low, indicating that medical personnel can effectively build interpersonal relationships with patients and treat them sincerely and warmly. This is consistent with the above finding regarding their generally positive attitude towards NM. Nevertheless, the mean scores for “I read disease-related narrative texts” (2.23) and “I try to write “medical confession stories” to alleviate my guilt about medical errors” (2.40) were relatively high, suggesting that most Chinese medical personnel relatively infrequently read or wrote narrative stories. This practice might be improved by providing systematic training courses that teach narrative skills and by establishing a platform that medical personnel can use to share their feelings and experiences concerning the reading and writing processes of NM.

Although the scoring rates of doctors alone were lower than those of all the participants numerically, there were no statistical significance identified, which indicates they may have some difficulties regarding NM in common.

### 4.2. Potential Influencing Factors for Knowledge, Attitude, and Practice regarding Narrative Medicine

Regression analyses revealed that working years is significant predictive factors for medical personnel's KAP. Longer working years predicts better knowledge, more positive attitude, and better practice, which is always accompanied by greater experience of listening to patients' stories, greater interaction with patients (and with a wider range of patients), and greater internalization of the relationship competencies learned in clinical practice [19, 20]. Moreover, younger doctors generally have a greater economic pressure to support their families out of their medical practice. Most of our participants are doctors working in public hospitals in China where the consultation fees for each patient is fix and relatively low, forcing these doctors, especially those who are younger, to see more patients during their limited outpatient time. This was also embodied in that medical personnel working in private medical institutions grasped more narrative knowledge and performed better narrative practice than their counterparts in public hospitals. However, considering the unbalanced structure of medical personnel working in different types of medical institutions, the generalization of this finding needs to be cautious. Meanwhile, education level and professional role were found to be influencing factors for both knowledge and attitude, which suggests that education level and professional role are inherently connected. One possible reason for this finding is the fact that doctors generally have higher education levels than other medical personnel. NM may be difficult to learn, and there is a risk that, when practicing NM, medical professionals will, as a result of the cognitive load, disregard other important parts of caring and healing [5]. Thus, medical personnel with higher education levels may have certain advantages in this regard, as they may be able to more easily comprehend and apply the key points of NM. Additionally, doctors, as a result of their daily work, naturally encounter more opportunities to apply narrative theory in communication with patients, which might also foster their narrative competence.

The article "Knowledge, Attitude, and Practice regarding Narrative Medicine among Chinese Medical Personnel: An Online Cross-Sectional Survey" was retracted in 2023. Reasons: signs of a paper mill; compromised peer review; unreliable results or conclusions.

Higher professional titles were found to be associated with better knowledge and practice, which may be attributed to such individuals' richer experience interacting with patients and reflecting on themselves. Further, professional titles may interact with the age factors of medical personnel, because those with higher professional titles generally have longer consultation time with each of their patients and less pressure about post promotion and family supporting [21], which could mean that they have more time to utilize narrative skills in their clinical practice. Time constraints can represent a major concern regarding the application of NM, as such constraints can limit the feasibility of shared doctor–patient decision-making [22, 23] and increase dissatisfaction on both sides [22–25]. Thus, greater efforts should be made to ensure medical staff have access to more clinical time.

Influencing factors of 836 doctors were identical to those of all the 2,145 medical personnel, which means the analyses performed above and the strategies formulated later may be suitable for physicians and surgeons, as well as other members of the medical system.

NM was not systematically introduced into China until 2011. During the subsequent 11 years, it has expanded in China mainly through three pathways: theoretical research, education for medical students, and clinical practice. However, such expansion has faced several obstacles, both external and internal [18]. On the one hand, although NM itself is still relatively novel, the theoretical system and discipline norms of NM have been weakly disseminated in China, which is reflected on that there have been few textbooks of NM in China. Approaches for training Chinese medical students differ from those used to train western students [26], and in China, medical humanities including NM are prone to be marginalized [26, 27] due to medical students' pressure for learning biomedical knowledge and getting good grades. Meanwhile, training of clinical professionals is mainly restricted to seminars and sessions, leaving insufficient time for them to master the focus skills or even experience the whole process of an approach. On the other hand, clinical medical staff in China are constantly busy, especially the younger ones who shoulder more pressure to make money and support their families, and, thus, do not have sufficient time to listen to their patients' stories in full, much less absorb or interpret these narratives. For example, a previous study analyzed 51 doctor–patient visits in an office setting and found that, on average, the doctors interrupted their patients just 18 seconds after the patients began to talk and that in only one of the 51 visits was the patient allowed to complete his/her narrative [28]. Additionally, there is currently a lack of appropriate systems, services, and support for NM; addressing this issue should be a priority for hospital, etc., administration, as this may mitigate frustration and demotivation among medical personnel.

The article "Knowledge, Attitude, and Practice regarding Narrative Medicine among Chinese Medical Personnel: An Online Cross-Sectional Survey" was retracted in 2023. Reasons: signs of a paper mill; compromised peer review; unreliable results or conclusions.

Thus, to support NM in China, both internal and external efforts are required. Compared with knowledge, Chinese medical personnel tended to have less satisfactory performance in narrative practice, indicating that they may be aware of the knowledge and importance of NM, but have difficulties in practice. This may due to challenges of three aspects: having no idea how to practice, why to practice, and having no time to practice. Future researchers should aim to establish and complete the theoretical system of NM and make the theories more accessible to medical personnel, which requires interdisciplinary collaboration of students, educators, and facilitators with different academic background, such as medicine-related subjects including clinical medicine, nursing, pharmacy, and traditional Chinese medicine, and humanities including literature, sociology, and ethics [13]. NM-related competence should be cultivated from the early stages of medical education (e.g., during training of undergraduate medical students and resident physicians, even when they study basic biomedical knowledge) and last for their whole career. However, the forms and contents of NM lessons are advised to be tailored according to their interests and worktime arrangement. For instance, literature of traditional Chinese medicine (TCM) may be an ideal but largely underexplored source of materials, especially for those majoring in or having interest in TCM [29]. Apart from lessons or seminars on NM, standardized “clinical guidelines” regarding NM are warranted for instruction and guidance in clinical settings. As for the problem of scant time for practice, relevant incentive and supporting measures which additionally target young physicians and surgeons should be adopted. Improving the treatment of younger doctors, especially those in public hospitals, can lessen their economic burdens and correct their tendency to receive more patients beyond ability, leaving more time for each patient and possibly facilitating narrative practice based on the NM-related knowledge doctors acquired before.

The article "Knowledge, Attitude, and Practice regarding Narrative Medicine among Chinese Medical Personnel: An Online Cross-Sectional Survey" was retracted in 2023. Reasons: signs of a paper mill; compromised peer review; unreliable results or conclusions.

Additionally, it may be beneficial to adopt a macroperspective in which more systematic, practical, and long-lasting narrative training is implemented. Since there has been limited literature on the long-term effect of NM on medical students and facilitators, large-scale promotion may start with pilot programs in several specific departments (e.g., oncology department and geriatrics department) in certain areas; and various new approaches could be tested. Studies have shown that on-site field practice and regular “sharing meetings” guided by NM professionals are generally more effective than traditional lectures [30]. Strategies may also be customized to suit the medical personnel's habits and the workflows of their specialty [31].

Overall, there has been great progress in the promotion of NM in China. As NM theory has gradually matured, the number of academic articles and textbooks focusing on NM in China has concurrently increased. Some medical schools are now offering NM-related options for senior medical students, and NM has also been included in resident training programs. Nevertheless, in the future, more targeted and long-lasting interventions aimed at expanding the application of NM theories are expected.

### 4.3. Limitations

Certain limitations to this online cross-sectional survey should be noted. First, as the questionnaire was distributed through an online survey platform and was mainly answered by medical personnel in urban areas (e.g., Beijing), our results may overrepresent Chinese medical personnel who are familiar with the Internet and who are located in metropolises. Thus, the generalizability of these findings is somewhat limited. Second, due to the particularity of NM, scales alone may not be sufficient to assess participants' KAP. Thus, further focus-group discussions and in-depth interviews are warranted. Third, we used a cross-sectional survey which has limited ability to infer causality. Fourth, certain questions (such as those about writing parallel medical records) may not be applicable to medical personnel except doctors although our results did not identify statistical differences. This incoherence of participants may affect the accuracy of our findings. Fifth, limitations on the length of and response times for online questionnaires mean that the list of influencing factors we identified might be incomplete. Future studies could expand our results by focusing on more doctors exclusively, incorporating open-ended questions with the measurement scales.

The article "Knowledge, Attitude, and Practice regarding Narrative Medicine among Chinese Medical Personnel: An Online Cross-Sectional Survey" was retracted in 2023. Reasons: signs of a paper mill; compromised peer review; unreliable results or conclusions.

## 5. Conclusion

With the aim of obtaining data that can help improve the prevalence and application of NM in China, this study preliminarily investigated Chinese medical personnel's KAP regarding NM and the factors that potentially influence this KAP. We consequently found that Chinese medical personnel's KAP regarding NM is generally positive, but that there remains scope for improvement. To advance the application of narrative skills in Chinese clinical practice, strategies based on theoretical, educational, and institutional perspectives should be applied. As the first study to explore the perception and usage of NM among national representatives of Chinese medical personnel, the present study provides practical insights into the development of NM in China. Limitations regarding the sample and the survey approach used mean further studies should aim for more demographic diversity among participants (and should especially target those in underdeveloped areas and medical students), compare the pre-post effect of NM education and practice, and combine quantitative analyses with qualitative analysis.

## Figures and Tables

**Table 1:** Basic information, univariate and multivariate analyses of factors associated with Chinese medical personnel's knowledge, attitude, and practice scores of narrative medicine (*N* = 2, 145).

Variable	*N* (%)	Knowledge (22.33 ± 4.87)				Attitude (23.42 ± 8.28)				Practice (24.84 ± 8.98)			
		*M* ± SD	*t*/*F*	*p*	*β*	*M* ± SD	*t*/*F*	*p*	*β*	*M* ± SD	*t*/*F*	*p*	*β*
Gender			0.436	0.509			0.309	0.579			0.035	0.851	
Female	931 (43.40)	22.41 ± 4.94				26.15 ± 6.41				24.88 ± 8.98			
Male	1214 (56.60)	22.27 ± 4.82				25.81 ± 6.64				24.81 ± 8.97			
Age			4.523	<0.001			5.087	<0.001			7.371	<0.001	
≤20	66 (3.08)	23.71 ± 4.92				28.58 ± 5.84				29.05 ± 9.07			
21-30	332 (15.48)	22.34 ± 4.67				25.50 ± 5.94				24.24 ± 8.66			
31-40	707 (32.96)	22.15 ± 4.90				26.18 ± 6.75				25.24 ± 9.39			
41-50	598 (27.88)	22.02 ± 5.05				25.93 ± 7.01				25.33 ± 9.26			
51-60	368 (17.16)	22.51 ± 4.72				25.67 ± 6.33				23.82 ± 8.24			
Other	74 (3.45)	24.39 ± 4.14				25.12 ± 3.53				21.16 ± 4.12			
Education level			9.819	<0.001	-0.118		5.301	<0.001	-0.069		9.757	<0.001	
Junior school and below	37 (1.72)	23.46 ± 4.27				29.51 ± 5.50				31.30 ± 7.75			
Senior school/technical secondary school	203 (9.46)	23.72 ± 4.08				27.04 ± 5.46				25.92 ± 8.44			
Associate degree	388 (18.09)	23.07 ± 4.93				26.86 ± 6.77				25.76 ± 9.59			
Undergraduate	874 (40.75)	21.83 ± 5.01				25.62 ± 6.87				24.83 ± 9.36			
Postgraduate and above	643 (29.98)	22.07 ± 4.78				25.32 ± 6.14				23.60 ± 8.00			
Marital status			15.457	<0.001			2.147	0.117			1.711	0.181	
Unmarried	355 (16.55)	22.66 ± 4.75				25.65 ± 5.74				24.28 ± 8.55			
Married	1,522 (70.96)	22.01 ± 4.95				25.90 ± 6.83				24.83 ± 9.20			
Divorced/widowed	268 (12.49)	23.73 ± 4.26				26.67 ± 5.75				25.63 ± 8.15			
Professional role			15.634	<0.001	0.042		7.078	<0.001	-0.008		10.673	<0.001	
Doctor	836 (38.97)	21.78 ± 4.81				25.69 ± 6.61				24.23 ± 8.73			
Pharmacist	411 (19.16)	23.10 ± 4.47				26.66 ± 5.78				25.49 ± 8.60			
Nurse	454 (21.17)	21.87 ± 4.80				25.01 ± 6.50				23.97 ± 8.47			
Technician	284 (13.24)	23.98 ± 4.86				28.09 ± 6.84				27.72 ± 10.62			
Manager	160 (7.46)	21.60 ± 5.48				24.44 ± 6.53				23.76 ± 8.27			
Professional title			11.982	<0.001	-0.058		13.306	<0.001			26.080	<0.001	-0.105
Primary	821 (38.28)	23.07 ± 4.88				27.46 ± 6.99				26.84 ± 10.08			
Intermediate	694 (32.35)	22.15 ± 4.82				25.61 ± 6.09				24.33 ± 8.38			
Associate senior	409 (19.07)	21.59 ± 4.72				24.39 ± 5.74				22.80 ± 7.28			
Senior	221 (10.30)	21.51 ± 4.92				24.36 ± 6.39				22.79 ± 7.66			
Working years			2.078	<0.001	-0.077		2.974	<0.001	-0.067		3.477	<0.001	-0.146
≤10	626 (29.18)	22.00 ± 5.03				26.20 ± 6.90				25.31 ± 10.06			
11~20	993 (46.29)	22.13 ± 5.02				26.75 ± 7.23				26.37 ± 10.02			
21~30	464 (21.64)	19.24 ± 3.94				22.44 ± 6.45				21.70 ± 7.08			
31~40	58 (2.70)	18.71 ± 4.05				21.22 ± 5.66				19.28 ± 5.72			
≥41	4 (0.19)	20.00 ± 4.97				24.00 ± 7.75				20.25 ± 3.69			
Institution categories			3.285	0.001	-0.071		1.288	0.198			2.424	0.015	-0.052
Public medical institutions	2,114 (98.55)	22.37 ± 4.87				23.44 ± 8.30				24.90 ± 8.99			
Private medical institutions	31 (1.45)	19.48 ± 4.42				21.52 ± 5.94				20.97 ± 6.82			

The article "Knowledge, Attitude, and Practice regarding Narrative Medicine among Chinese Medical Personnel: An Online Cross-Sectional Survey" was retracted in 2023. Reasons: signs of a paper mill; compromised peer review; unreliable results or conclusions.

**Table 2:** General cognition and basic knowledge of narrative medicine among 2,145 Chinese medical personnel.

Dimension	Item	Option	*N* (%)
General cognition	Understanding of NM	Never heard	423 (19.72)
		Not very familiar, only heard or browsed	729 (33.99)
		Relatively familiar, know its concept	635 (29.60)
		Very familiar, have participated in some systematic trainings	358 (16.69)
	Pathways to understanding NM	Lectures	780 (41.85)
		Internet	908 (48.71)
		Conferences	892 (47.85)
		Textbooks	674 (36.16)
		Training courses	737 (39.54)
		Journals	480 (25.75)
		Others^∗^	24 (1.29)
	Understanding of parallel medical records	Never heard	512 (23.87)
		Not very familiar, only heard or browsed	737 (34.36)
		Relatively familiar, know its concept	578 (26.95)
		Very familiar, have participated in some systematic trainings	318 (14.83)
	Ever practice of NM-related skills in daily work	Yes	1,167 (54.41)
		No	978 (45.59)

Basic knowledge	Ability to distinguish between “disease” and “sickness”	No, I cannot.	514 (23.96)
		Yes, I can. The former is the doctors' world of and the latter is the patients' world.	1,631 (76.04)
	Contents of narrative relationship in medical field	Doctors and patients	1,497 (69.79)
		Doctors and themselves	1,314 (61.26)
		Doctors and their colleagues	1,530 (71.33)
		Doctors and society	1,236 (57.62)
	Contents of narrative types	Patients' stories	1,477 (68.86)
		Doctors' stories	1,290 (60.14)
		Narratives of doctor-patient contact	1,661 (77.44)
		Grand narratives (metanarratives)	911 (42.47)
	Narrative types which parallel medical records belong to	Patients' stories	552 (25.73)
		Doctors' stories	447 (20.84)
		Narratives of doctor-patient contact	783 (36.50)
		Grand narratives (metanarratives)	363 (16.92)

Note: NM = narrative medicine; ^∗^ included communicating with others, recommendation from colleagues, WeChat (e.g., moments and official accounts), reading relevant works (especially Rita Charon's works), and participating in the compilation of NM textbooks.

**Table 3:** Knowledge scores of Chinese medical personnel on narrative medicine (*N* = 2, 145).

Item	Option										*M* ± SD
	Strongly agree		Relatively agree		Uncertain		Relatively disagree		Strongly disagree		
	Score	*N* (%)	Score	*N* (%)	Score	*N* (%)	Score	*N* (%)	Score	*N* (%)	
(16) NM embodies the concept of patient-centered medicine.	1	835 (38.93)	2	724 (33.75)	3	332 (15.48)	4	137 (6.39)	5	117 (5.45)	2.06 ± 1.14
(15) NM involves applying literary theories to medical practice.	1	739 (34.45)	2	742 (34.59)	3	436 (20.33)	4	124 (5.78)	5	104 (4.85)	2.12 ± 1.10
(29) NM advocates paying attention to both patients' and doctors' negative emotions.	1	749 (34.92)	2	719 (33.52)	3	398 (18.55)	4	175 (8.16)	5	104 (4.85)	2.14 ± 1.13
(20) Empathy with patients is one of the focuses of NM.	1	660 (30.77)	2	805 (37.53)	3	373 (17.39)	4	182 (8.48)	5	125 (5.83)	2.21 ± 1.14
(19) Doctors should encourage patients to tell their stories to get information about their condition.	1	710 (33.10)	2	756 (35.24)	3	340 (15.85)	4	195 (9.09)	5	144 (6.71)	2.21 ± 1.19
(23) Through reflective writing, we can realize the “reproduction” in NM.	1	681 (31.75)	2	748 (34.87)	3	406 (18.93)	4	156 (7.27)	5	154 (7.18)	2.23 ± 1.18
(22) Close reading and reflective writing are two tools of NM.	1	677 (31.56)	2	730 (34.03)	3	431 (20.09)	4	170 (7.93)	5	137 (6.39)	2.24 ± 1.16
(21) The most important purpose of NM is to establish relationship, which only refers to the doctor-patient relationship.	5	521 (24.29)	4	681 (31.75)	3	458 (21.35)	2	312 (14.55)	1	173 (8.07)	3.50 ± 1.23
(18) Shared decision-making among doctors and patients is not a practical way of implementing NM.	5	607 (28.30)	4	663 (30.91)	3	469 (21.86)	2	272 (12.68)	1	134 (6.25)	3.62 ± 1.20

Note: NM = narrative medicine.

The article "Knowledge, Attitude, and Practice regarding Narrative Medicine among Chinese Medical Personnel: An Online Cross-Sectional Survey" was retracted in 2023. Reasons: signs of a paper mill; compromised peer review; unreliable results or conclusions.

**Table 4:** Attitude scores of Chinese medical personnel on narrative medicine (*N* = 2, 145).

Item	Option										*M* ± SD
	Strongly agree		Relatively agree		Uncertain		Relatively disagree		Strongly disagree		
	Score	*N* (%)	Score	*N* (%)	Score	*N* (%)	Score	*N* (%)	Score	*N* (%)	
(39) I am willing to study NM-related courses.	1	845 (39.39)	2	669 (31.19)	3	425 (19.81)	4	123 (5.73)	5	83 (3.87)	2.03 ± 1.08
(34) I think cultivating narrative ability can improve my attention and understanding of patients and enhance humanistic care.	1	771 (35.94)	2	771 (35.94)	3	401 (18.69)	4	106 (4.94)	5	96 (4.48)	2.06 ± 1.07
(31) I think an NM approach can provide patients with more personalized, humanized, and effective treatment.	1	821 (38.28)	2	694 (32.35)	3	408 (19.02)	4	121 (5.64)	5	101 (4.71)	2.06 ± 1.10
(38) I think understanding the patients' stories will help me to reunderstand my stories and life value.	1	818 (38.14)	2	698 (32.54)	3	393 (18.32)	4	132 (6.15)	5	104 (4.85)	2.07 ± 1.12
(37) I am willing to narrate my medical practice and patients' stories and share them with my colleagues or the public.	1	809 (37.72)	2	678 (31.61)	3	437 (20.37)	4	125 (5.83)	5	96 (4.48)	2.08 ± 1.10
(36) NM can improve my communication skills and help me maintain a good relationship with patients and their families.	1	774 (36.08)	2	756 (35.24)	3	381 (17.76)	4	136 (6.34)	5	98 (4.57)	2.08 ± 1.09
(35) I think NM can improve my working experience and professional identity.	1	803 (37.44)	2	695 (32.4)	3	414 (19.3)	4	117 (5.45)	5	116 (5.41)	2.09 ± 1.13
(40) I hope to spread the methods of NM in clinical practice.	1	801 (37.34)	2	672 (31.33)	3	441 (20.56)	4	135 (6.29)	5	96 (4.48)	2.09 ± 1.11
(30) I think NM can improve patients' medical experience and ease the doctor-patient relationship.	1	737 (34.36)	2	764 (35.62)	3	406 (18.93)	4	130 (6.06)	5	108 (5.03)	2.12 ± 1.10
(33) I do not think parallel medical records can help me better treat patients, but increase my workload.	5	670 (31.24)	4	537 (25.03)	3	517 (24.1)	2	276 (12.87)	1	145 (6.76)	3.61 ± 1.24
(32) I do not think practicing NM will have any effect on my medical practice.	5	682 (31.79)	4	562 (26.2)	3	510 (23.78)	2	268 (12.49)	1	123 (5.73)	3.66 ± 1.21

Note: NM = narrative medicine.

The article "Knowledge, Attitude, and Practice regarding Narrative Medicine among Chinese Medical Personnel: An Online Cross-Sectional Survey" was retracted in 2023. Reasons: signs of a paper mill; compromised peer review; unreliable results or conclusions.

**Table 5:** Practice scores of Chinese medical personnel on narrative medicine (*N* = 2, 145).

Item	Option										*M* ± SD
	Always		Occasionally		Uncertain		Seldom		Never		
	Score	*N* (%)	Score	*N* (%)	Score	*N* (%)	Score	*N* (%)	Score	*N* (%)	
(41) I am able to maintain good relationships with the patients I meet in my daily work.	1	1,060 (49.42)	2	523 (24.38)	3	338 (15.76)	4	130 (6.06)	5	94 (4.38)	1.92 ± 1.13
(50) I have sincere discussions with patients on a daily basis.	1	964 (44.94)	2	620 (28.9)	3	356 (16.6)	4	113 (5.27)	5	92 (4.29)	1.95 ± 1.10
(42) I listen carefully to the patients about things not related to their symptoms (occupation, interpersonal relationships, difficulties, wishes, their views of the disease, etc.) in my daily work.	1	979 (45.64)	2	585 (27.27)	3	370 (17.25)	4	118 (5.5)	5	93 (4.34)	1.96 ± 1.11
(44) I can detect the changes in the patients' moods and behaviors and respond appropriately in my daily work.	1	977 (45.55)	2	571 (26.62)	3	376 (17.53)	4	126 (5.87)	5	95 (4.43)	1.97 ± 1.12
(49) I reflect on the process of clinical diagnosis and treatment activities.	1	929 (43.31)	2	641 (29.88)	3	350 (16.32)	4	128 (5.97)	5	97 (4.52)	1.99 ± 1.12
(43) I take the initiative to care about patients' personal life without violating privacy in my daily work.	1	889 (41.45)	2	652 (30.4)	3	357 (16.64)	4	152 (7.09)	5	95 (4.43)	2.03 ± 1.12
(48) I try to empathize with the patients' painful experience in my daily work.	1	834 (38.88)	2	667 (31.1)	3	390 (18.18)	4	157 (7.32)	5	97 (4.52)	2.08 ± 1.13
(51) I invite patients and their families to participate in medical decision-making and ask them to express their thoughts, concerns, and expectations in my daily work.	1	829 (38.65)	2	670 (31.24)	3	374 (17.44)	4	165 (7.69)	5	107 (4.99)	2.09 ± 1.14
(52) I read NM-related stories written by my colleagues.	1	738 (34.41)	2	756 (35.24)	3	417 (19.44)	4	132 (6.15)	5	102 (4.76)	2.12 ± 1.10
(45) Patients are willing to tell me about their thoughts and more personal things in my daily work.	1	750 (34.97)	2	750 (34.97)	3	384 (17.9)	4	151 (7.04)	5	110 (5.13)	2.12 ± 1.12
(46) I read disease-narrative texts in my life.	1	651 (30.35)	2	743 (34.64)	3	466 (21.72)	4	181 (8.44)	5	104 (4.85)	2.23 ± 1.12
(47) I try to write “medical confession stories” to alleviate my guilt regarding medical errors.	1	660 (30.77)	2	574 (26.76)	3	487 (22.7)	4	234 (10.91)	5	190 (8.86)	2.40 ± 1.27

Note: NM = narrative medicine.

The article "Knowledge, Attitude, and Practice regarding Narrative Medicine among Chinese Medical Personnel: An Online Cross-Sectional Survey" was retracted in 2023. Reasons: signs of a paper mill; compromised peer review; unreliable results or conclusions.

## Data Availability

The data generated and analyzed during the current study are not publicly available due to the participants' privacy but are available from Yongli Sun (yonglisunlove@ccmu.edu.cn) for any questions or requests.

## Supplementary Materials

Supplementary Materials Supplementary Table 1: basic information, univariate and multivariate analyses of factors associated with 836 Chinese doctors' knowledge, attitude and practice scores of narrative medicine. Supplementary Table 2: general cognition and basic knowledge of narrative medicine among 836 Chinese doctors. Supplementary Table 3: knowledge scores of 836 Chinese doctors on narrative medicine. Supplementary Table 4: attitude scores of 836 Chinese doctors on narrative medicine. Supplementary Table 5: practice scores of 836 Chinese doctors on narrative medicine.
